# MiR-125b-5p/STAT3 Axis Regulates Drug Resistance in Osteosarcoma Cells by Acting on ABC Transporters

This article has been retracted.

**DOI:** 10.1155/2023/9997676

**Published:** 2023-04-29

**Authors:** Yang Yang, Yueyuan Chen, Jiajia Liu, Bo Zhang, Linlin Yang, Jianhua Xue, Zexu Zhang, Lili Qin, Rongpeng Bian

**Affiliations:** ^1^Department of Trauma Center, Affiliated Hospital of Nantong University, Nantong City, Jiangsu Province 226001, China; ^2^Department of Oncology, Second People's Hospital of Nantong, Nantong City, 226001 Jiangsu Province, China; ^3^Department of Orthopaedics, Affiliated Hospital of Nantong University, Nantong City, Jiangsu Province 226001, China; ^4^Department of Oncology, Sheyang People's Hospital, Yancheng City, Jiangsu Province 224300, China; ^5^Department of Endoscopic Center, Affiliated Hospital of Nantong University, Nantong City, Jiangsu Province 226001, China; ^6^Department of Orthopedic Surgery, The Fourth Affiliated Hospital of Nantong University, Yancheng City, Jiangsu Province 224000, China; ^7^Department of Orthopedic Surgery, The First People's Hospital of Yancheng, Yancheng City, Jiangsu Province 224000, China

## Abstract

**Background:**

The poor prognosis of the highly malignant tumor osteosarcoma stems from its drug resistance and therefore exploring its resistance mechanisms will help us identify more effective treatment options. However, the effects of miR-125b-5p on drug resistance in osteosarcoma cells are still unclear.

**Methods:**

To study the effects of miR-125b-5p on drug resistance in osteosarcoma cells. Osteosarcoma-resistant miR-125b-5p was obtained from the databases GeneCards and g:Profiler. CCK8, western blot, and transwell were applied for the detection of the miR-125b-5p effects on proliferation, migration, invasion, apoptosis, and drug resistance in osteosarcoma. Bioinformatics is aimed at demonstrating the targeting factor miR-125b-5p, performing protein interaction enrichment analysis by Metascape, and finally validating by binding sites.

**Results:**

Upregulation of miR-125b-5p restrains proliferation, migration, and invasion of osteosarcoma and promotes apoptosis. In addition, miR-125b-5p can restore drug sensitivity in drug-resistant osteosarcoma. miR-125-5p restrains the signal transducer and inhibits the transcription 3 (STAT3) expression activator via targeting its 3′-UTR. STAT3 affects drug-resistant osteosarcoma to regulate the ABC transporter.

**Conclusion:**

miR-125b-5p/STAT3 axis mediates the drug resistance of osteosarcoma by acting on ABC transporter.

## 1. Introduction

Osteosarcoma (OSA), as a primary bone malignant tumor, is characterized by pathology and frequent distant metastases, leading to youth death worldwide [1]. Patients with local OSA usually have 60-80% of 5-year survivals. For sufferers with recurrent or metastatic disease, the 5-year survival rate is reduced to 15-30% [2, 3]. The potential targets have been developed for OSA treatment by the latest advances in bioinformatics and technology [4–6]. Therefore, there is an urgent need to find a key metastasis-related molecule and determine its potential mechanism in OSA. Uncovering the underlying mechanisms that determine the chemosensitivity and resistance of OSA seems crucial. OSA is an allogeneic disease characterized by a high degree of genome instability, extensive genetic aberrations, and a variety of disturbed signaling pathways. OSA is classified into low-, intermediate-, and high-grade tumors histopathologically according to the grade of differentiation. High-grade osteosarcomas (HGOS) account for almost 90% among OSAs and are further subclassified into telangiectatic, conventional, small-cell, surface, and secondary tumors [7]. OSA is particularly resistant to chemotherapy. These tumors only respond to high-dose chemotherapy and quickly acquire drug resistance. This is reflected in the low rescue rate: only 20% of recurrent patients survived [8].

Chemical resistance remains a huge obstacle encountered in OSA treatment [9]. MicroRNAs (miRNAs) partake in specific complementation and binding for a target gene to the 3′-untranslated region (UTR). In many cellular processes, miRNAs have critical functions in regulating posttranscriptional gene expression, including fate determination and cell differentiation. In addition, they also play vital roles in the chemical resistance of tumors [10, 11]. miR-582-5p restrains OSA cell growth and invasion via targeting NOVA1 [12]. LINC01410 sponges miR-3128 to accelerate OSA invasion and proliferation [13]. Previous study has shown that miR-125b-5p sponge to mediate the tumorigenicity, which could act as a potential biomarker for the osteosarcoma and provides a novel insight for the mechanism in osteosarcoma [14]. Nevertheless, the underlying mechanism of miRNAs regulating inflammation and regeneration is obscure. It has been reported that some important messenger RNA (mRNA) and noncoding RNAs (ncRNA) are involved in OSA chemotherapy resistance, including resistance to MTX, miR-33a and DDP resistance of RFC, and lncRNA FOXC2-AS1 resistance to DXR [15, 16].

Multidrug resistance (MDR) is recognized as the main factor of chemotherapeutic failure in OSA [17]. The molecular mechanisms include attenuation of intracellular drug concentration through enhanced DNA repair and activating the drug efflux pump [18].

The ABC superfamily is a transport protein family with 49 members, according to its sequence and structure. As a glycosylated 170-kDa transmembrane protein [19], ABCB1 (P-glycoprotein/MDR1) is known as a principal reason for resistance in various cancers [20]. Its upregulation in cancers conduces to a reduction of intracellular chemotherapeutic accumulation and leads to antineoplastic drug resistance.

Signal transducers and activators of transcription (STAT) proteins are significant transcriptional factors as latent cytoplasmic transcription factors, involving in proliferation, survival, apoptosis, angiogenesis, and metastasis of tumor [21]. STAT3 is expressed widely and transiently activated responding to interleukin-6 (IL-6) and epidermal growth factor (EGF) by tyrosine phosphorylation [22]. Overexpressed STAT3 is implicated in OSA development, progression, and bad prognosis. STAT3 has been accepted as a latent key therapeutic target for OSA [23]. Known as acute-phase response factor (APRF), the STAT3 protein consists of other six domains: the DNA binding domain, Src homology 2 (SH2) domain, a coiled-coil domain, an amino-terminus, a carboxyterminal transactivation domain, and a linker domain [24]. STAT3 is activated in different cancer types, such as lung cancer, breast cancer, and ovarian cancer [25]. Thus, we propose a hypothesis that miR-125b-5p might regulate drug resistance in osteosarcoma cells through STAT3 by acting on ABC transporters.

## 2. Materials and Methods

### 2.1. Materials

U-20S/DX580 and Sao-2/DX580 cell lines were acquired from the Chinese Academy of Sciences Cell Bank (Shanghai, China) and preserved with DMEM and DMEM/F12 (Gibco, El Paso, TX, USA), respectively. All mediums contained streptomycin 100 mg/mL (Baomanbio, China), penicillin 100 IU/mL (Baomanbio, China), and 10% (*v*/*v*) fetal bovine serum (FBS, Sigma, St. Louis, MO, USA). All OSA cell lines were fostered at 37°C in a damp condition including 5% CO_2_.

### 2.2. Cell Transfection

Briefly, U-20S/DX580 and Sao-2/DX580 cells at 1 × 10^6^ cells/ml were plated in a 6- or 24-hole plates and then, respectively, transfected with 100 nmol/l miR-125b-5p mimic (Shanghai GenePharma Co., Ltd.), or miR-125b-5p mimic control vector (Shanghai GenePharma Co., Ltd.) in a mixture with Lipofectamine® 3000 (L3000015; Thermo Fisher Scientific, Inc.) and 2.5 *μ*g/*μ*l SonoVue microbubbles (Bracco Suisse SA) under the irradiation of ultrasonic transfer apparatus via ultrasound couplant (Anhui Deepblue Medical Technology Co., Ltd.) at the parameters of 0.5 W/cm2 for 30 sec. The cells in the L group were transfected with miR-125b-5p mimic using Lipofectamine 3000 only, while those in the Blank group were treated with medium only. All the cells were cultured for another 72 h after the transfection.

### 2.3. Animals

We performed experiments using Sprague–Dawley rats (7-8 week old; male; 200–220 g) from the Laboratory Animal Center of Nantong University. Raised the rats in constant-temperature plastic chambers (25°C) and offered food and water, with a light–dark cycle lasting for 12 h starting at 8 : 00 am.

### 2.4. Reagents

Antibodies were supplied by Proteintech (Wuhan, China), Cell Signaling Technology (Beverly, MA, USA), and Abcam (Cambridge, UK). RiboBio (Guangzhou, China) was used to synthesize inhibitors, miminc, primers, and their respective NCs. Fetal bovine serum, DMEM, penicillin–streptomycin, and phosphate-buffered saline were provided by Gibco. High purity was used for other reagents.

### 2.5. RT-qPCR

With TRIzol® Reagent (Invitrogen, Carlsbad, CA, USA), isolated total RNA from cultured cells accordingly. Then cDNA was synthesized by the RevertAid™ First Strand cDNA Synthesis Kit (Thermo Scientific, Waltham, MA, USA). Used gene-specific primers to conduct real-time RT-qPCR by SYBR® Premix Ex Taq™ (Bio-Rad Laboratories) and adopted 2^−*ΔΔ*CT^ method [26] to determine relative miRNA and mRNA expressions and normalized to U6 or *β*-actin expression. The primers were as follows: miR-125b-5p forward, 5′-ACACTCCAGCT GGGTCCCTGAGACCCTAAC-3′, and reverse, 5′-CTCAAC TGGTGTCGTGGAGTCGGCAATTCAGTTGA-3′; U6 forward, 5′-CTCGCTTCGGCAGCACA-3′, and reverse, 5′-AACGCTTCACGAATTTGCG-3′; *β*-actin forward, 5′-TCCCTGGAGAAGAGCTACGA-3′, and reverse, 5′-AGCACTGTGTTGGCGTACAG-3′; STAT3 forward, 5′-CAGGAGGGCAGTTTGAGTCC-3′, and reverse, 5′-CAAAGATAGCAGAAGTAGGAGA-3′.

### 2.6. Cell Counting Kit (CCK)-8 Assay

Cell viability evaluation was conducted using the CCK-8 (Biosharp) assay. U-20S/DX580 cells were treated by transfection of miR-125b-5p mimic or NC mimics and later fostered in 96-hole plates at 1 × 10^5^ cells/mL. After 24, 48, and 72 h, DMEM supplementary with 10% CCK-8 was added for a 2 h incubation. Subsequently, used a microplate reader to measure the absorbance.

### 2.7. Western Blotting

Samples were abstracted with RIPA buffer (Biosharp, Hefei, China). With a bicinchoninic acid protein assay kit (Biosharp, Hefei, China), the protein concentration was accessed. The supernatant was added with sodium dodecyl sulfate-polyacrylamide electrophoresis (SDS-PAGE) loading buffer (Beyotime, Shanghai, China) and heated at 95°C for 10 min. Protein samples (30 *μ*g) were transferred onto 0.2 or 0.45 *μ*m polyvinylidene fluoride (PVDF) membranes (Millipore, Bedford, MA, USA) with 12% Tris-glycine gels (Epizyme, Shanghai, China), sealed in 5% skimmed milk (Sangon Biotech, Shanghai, China), and then kept overnight at 4°C with primary antibodies. The next day, 1 h of room temperature incubation for the membranes with secondary antibodies and protein bands detection on X-ray film by enhanced chemiluminescence detection system.

### 2.8. Wound-Healing Migration Assay

For wound-healing assays, U-20S/DX580 and Saoa-2/DX580 cells were treated with culture medium after being inoculated onto six-hole plates at 70% confluence and then transfected with NC mimics or miR-125b-5p mimic. Around 48 h later, scratched fused cell monolayer using a fine pipette tip and observe the wound closure rate at the indicated times with a microscope.

### 2.9. Dual Luciferase Reporter Assay

To clarify the association of STAT-3 with miR-125b-5p, the following experiment was performed. First, U-20S/DX580 and Saoa-2/DX580 cells were inoculated into 24-hole plates and cotransfected on a shaking platform for 24 h by mimics NC, mimics, psi-CHECK2-STAT-3 WT vector, and psi-CHECK2- STAT-3 Mut vector after 15 min lysis with Passive Lysis Buffer (30 mL, Promega, Fitchburg, WI, USA), followed by measurement of dual-luciferase activity [27].

### 2.10. Flow Cytometry

After transfection for 48 hours, washed the cells in 0.01 mol/L PBS, removed the supernatant, centrifuged for 5 min at 2500 g, suspended in 1× binding buffer, and adjusted to 1 × 10^6^ cells/mL. Each tube was added with cell suspension 500 *μ*L, propidium iodide 10 *μ*L, and Annexin V-fluorescein isothiocyanate 5 *μ*L (Invitrogen Inc., Carlsbad, CA, USA), mixed, kept for 10 mins at room temperature, and finally detected by flow cytometer.

### 2.11. Statistical Analysis

Mean ± standard deviation was used for data expression and Prism 9 (GraphPad, San Diego, CA, USA) for data analysis. Student's t-test, one-way analysis of variance, and Tukey's post hoc test were applied to analyze statistical discrepancy between groups. *P* < 0.05 means statistically significant.

## 3. Result

### 3.1. miR-125-5p Expression in OSA Tissues and Cell Lines

Five miRNAs (miR-155-5p, miR-18a-5p, miR-451a, miR-145-3p, and miR-125-5p) were found in predictive software. Among them, miR-125-5p has the highest expression level (Figure 1(a)). Next, the expression of miR-125-5p was decreased significantly in tumor tissues (Figure 1(b)). To further study the action mechanism of miR-125-5p in OSA, expression of miR-125-5p in OSA cell lines (U-20S, U-20S/DX580 and SaOS-2, Sao-2/DX580) were detected (Figure 1(c)), and U-20S/DX580 and Sao-2/DX580 cells with high miR-125-5p expression were screened in subsequent experiments.

### 3.2. Affection of High miR-125b-5p Expression on the Invasion, Proliferation, and Migration of Drug-Resistant OSA

Compared to the negative control group, the miR-125b-5p mimic group showed obviously increased expression of miR-125-5p after transfection (Figure 2(a)). The CCK-8 assay illustrated that different mimic treatment time affected cell viability. In the miR-125-5p mimic group, the cell viability was obviously decreased in U-20S/DX580 and Sao-2/DX580 cells (Figure 2(b)). Results of western blot revealed that CDK2 and cyclinE1 protein were declined significantly in miR-125-5p mimics group (*P* < 0.01) (Figures 2(b) and 2(c)), and protein p21 was ascend significantly (Figure 2(c)). Results of the scratch assay and transwell assay suggested that miR-125-5p mimic slowed down migration in U-20S/DX580 and Sao-2/DX580 cells (Figure 2(d)). MMP2 and MMP9 protein expression was also identified by western blot and discovered to be decreased significantly in miR-125-5p mimic group after cell transfection compared with that in the mimic NC group (Figure 2(f)).

### 3.3. High miR-125b-5p Expression Enhances the Sensitivity of Drug-Resistant OSA

Cell viability was discovered to be affected by the different doses of drug therapy by the CCK-8 assay (Figure 3(a). Cell overexpressing miR-125-5p had lower viability than NC cells. Overexpression of miR-125-5p remarkably increased the apoptotic rate in U-20S/DX580 and Sao-2/DX580 cells (Figure 3(b)) compared with the control group by flow cytometric analysis. Furthermore, western blot revealed that active caspase-3 protein and Bax protein elevated significantly in the miR-123-5p mimic group, while the Bcl-2 protein was decreased.

### 3.4. miR-125-5p Restrains STAT3 Expression via Targeting Its 3'-UTR

Compared to the NC mimic group, the luciferase activity of the psi-CHECK2-STAT-3 WT vector was significantly decreased in the miR-125-5p mimic group. However, the STAT3-MuT group showed no significant changes in both in U-20S/DX580 and Sao-2/DX580 cells. Combined with the results of sequencing and prediction, STAT appeared to be a molecular target of miR-125-5p (Figures 4(a) and 4(b)). Compared to the NC mimic group, the expression of STAT3 in the miR-125-5p mimic group declined to a certain level (Figure 4(c)). A western blot was conducted to further confirm the results (Figure 4(d)). Finally, we concluded that STAT3 acts as a biological target of miR-123-5p.

### 3.5. STAT3 Restores Tumor Resistance by Regulating ABC Transporter

In tumor tissues, the expression of STAT3 was significantly increased (Figure 5(a)). For further study on the role of STAT3 in OSA, expression of STAT3 in OSA cell lines (U-20S, U-20S/DX580, SaOS-2, and Sao-2/DX580) was detected (Figure 5(b)), and U-20S/DX580 and Sao-2/DX580 with high miR-125-5p expression were collected for follow-up experiments. To figure out the relationship between STAT3 and ABC in U-20S/DX580 and Sao-2/DX580, the expression of STAT3 was knocked down by inserting specific small interfering RNA (sh-STAT3). After transfection with sh-STAT3 for 24 h, western blot revealed that sh-STAT3 could effectively decrease the expression of ABCB1 and ABCC1 (Figure 5(c)).

### 3.6. STAT3 Reversed the Sensitivity of Drug-Resistant OSA

The CCK-8 assay implied that different doses of drug treatment affected cell viability. Artificially increasing the level of STAT reversed miR-125-5p function on drug-resistant OSA. Additionally, treating with Pc-STAT3 and miR-125-5p could increase the cell viability of U-20S/DX580 and Sao-2/DX580 compared with that using miR-125-5p mimic and pc-NC, which means that the effect of miR-125-5p to inhibit tumor cell drug resistance is removed by STAT3 (Figure 6(a)). The same result appears in apoptosis-related protein expression. The results suggested that the decreased expression of Bax and active Caspase-3 was due to increased expression of miR-125-5p, but after the additional treatment of pc-STAT3, this down trend was reversed, which means that high expression of STAT3 will reduce tumor cell apoptosis (Figure 6(b)).

## 4. Discussion

In our current research, we first revealed significantly decreased miR-125-5p expression in OSA tissues. Then it was proven that miRNA overexpression can inhibit OSA proliferation, invasion, and migration. In addition, miRNAs can also restore the drug sensitivity of drug-resistant OSA. Through bioinformatics and experiments, we predicted the downstream target between miRNAs and STAT3 and verified that miR-125-5p suppresses STAT3 expression via targeting its 3′-UTR. Then, it was verified that STAT3 regulates the ABC transporter to affect drug-resistant OSA. Finally, we proved that the miR-125b-5p/STAT3 axis regulates drug resistance in OSA by acting on the ABC transporter.

To this day, miRNAs have been participated in almost all aspects of biological processes and cell functions. miRNAs are expressed abnormally in diverse cancers and have a close relationship to invasion, metastasis, and proliferation [28–30]. Therefore, a better understanding of microRNAs may provide different perspectives on oncogenesis and promote treatment for cancer treatment. LncRNA SNHG6/miR-125b-5p/BMPR1B Axis was demonstrated as a novel therapy direction for triple-negative breast cancer [31]. Extracellular vesicles derived from tumors have the potential to carry the miR-125b-5p target TNFAIP3, which can reduce the sensitivity of diffuse large B cell lymphoma to rituximab [32]. CircVAPA advances malignant progression and chemotherapy resistance in gastric cancer via miR-125b-5p/STAT3 signaling [33]. Circular RNA 0086996 mediates OSA cell migration and growth via miR-125b-5p [14]. The mTORC1-regulated miR-125b-5p/STAT3 pathway exerts a significant role in promoting tumor growth and cell proliferation [34]. A lot of discussions about miR-125b-5p have been performed; however, there have been few investigations on the drug-resistant OSA role of miR-125b-5p. We also found that miRNA overexpression can inhibit OSA migration, proliferation, and invasion. Furthermore, miRNAs can also restore the drug sensitivity of drug-resistant OSA. Through bioinformatics and experiments, we predicted and verified the downstream target between miR and STAT3. Our findings indicate that STAT3 regulates ABC transporter to affect drug-resistant OSA and finally proved that the miR-125b-5p/STAT3 axis modulates the drug resistance of OSA by acting on ABC transporter. SH003 reverts drug resistance by blocking STAT3 signaling in breast cancer cells [35].

STAT family, including STAT1-5 and STAT6, are vital transducers of many growth factors and cytokines (ILs). STAT3 is overexpressed or activated constitutively in tumors compared with normal tissue [22]. Excessive STAT3 activation within cancer cells can be viewed as an attractive target for cancer therapy [36]. Cisplatin resistance can be reduced by a ferrocene derivative in breast cancer cells through modulating JAK2/STAT3 pathway and suppressing MDR-1 expression [37]. ATP-binding cassette transporters were independently regulated by STAT3 in the chemoresistance of gastric cancer cells [38]. LncRNA-MALAT1 upregulates MDR1 and MRP1 through STAT3 activation to contribute to the cisplatin resistance of lung cancer [39]. We further revealed that increasing STAT expression reverses the effect of miR-125-5p on drug resistance in OSA. However, this down trend was reversed after the additional treatment of pc-STAT3, which means that high expression of STAT3 will reduce tumor cell apoptosis. Our results are consistent with the previous conclusions to some extent.

ATP-binding cassette transporter B1 (ABCB1) promotes chemoresistance in OSA because it can release doxorubicin, thereby reducing immunogenic cell death, drug-induced intracellular toxicity, and accumulation. We knocked down STAT3 expression through the introduction of specific small interfering RNA (sh-STAT3). After transfection with sh-STAT3 for 24 h, western blot revealed that sh-STAT3 could effectively decrease ABCB1 and ABCC1 expressions. Which means STAT3 can restore tumor resistance by regulating the ABC transporter. Although we discovered that miR-125b-5p/STAT3 axis modulates the drug resistance of OSA cells by acting on ABC transporters, we cannot exclude the possibility that the miRNA overexpression may show its resistance to OSA through other signaling pathways. Therefore, further research is needed to more comprehensively reveal the molecular mechanism of its resistance to OSA.

## 5. Conclusion

To sum up, our results revealed the miR-125b-5p/STAT3 axis modulates drug resistance of OSA by acting on the ABC transporter.

## Figures and Tables

**Figure 1:** Screening and prediction of miR-125-5p. (a) Among the five predicted miRNAs, miR-125-5p had the highest expression. The horizontal coordinate represents the -log10 (adjusted *P* value), and the vertical coordinate represents the 5 miRNAs screened. (b) miR-125-5p expression in osteosarcoma (OSA) and normal samples. The vertical coordinate represents the relative expression quantity. miR-125b-5p is less expressed in OSA than in normal tissue. (c) miR-125-5p expression in four cell lines of OSA. The vertical coordinate represents the relative expression quantity. ^∗∗∗^represents *P* < 0.001.

**Figure 2:** miR-125-5p effect on proliferation, migration, and invasion of drug-resistant OSA. (a) Transfection efficiency of miR-125-5p after 24 hours. (b) CCK8 showed cell viability at different time periods of transfection (0, 24, 48, and 72 h). (c) Expression of cell cycle-associated proteins in two OSA cell lines transfected with miR-125-5p. (d) The scratch and transwell assays were designed to reflect cell migration ability after transfection with miR-125-5p. (e) metalloplasmin-related proteins are designed to reflect the invasive ability of cells after transfection with miR-125b-5p. ^∗^represents *P* < 0.05; ^∗∗^represents *P* < 0.01; ^∗∗∗^represents *P* < 0.001.

**Figure 3:** Effect of transfection with miR-125b-5p on cell viability and apoptosis. (a) Differences in cell viability after transfection with miR-125b-5p at different drug concentrations. (b) The flow cytometric analysis was designed to reflect apoptosis after transfection with miR-125b-5p. (c) Expression of apoptosis-associated proteins in OSA cell lines after transfection with miR-125b-5p. ^∗^represents *P* <0.05; ^∗∗^ represents *P* <0.01; ^∗∗∗^represents *P* < 0.001.

**Figure 4:** Prediction of molecular targets of miR-123-5p. (a, b) The expression of control cells and cells transfected with miR-125-5p in the predicted targets STAT3-WT and STAT3-Mut, which showed differences in STAT3-WT. (c) RT-qPCR for demonstrating STAT3 expression in cell lines transfected with miR-125-5p in OSA. (d) Western blot for demonstrating STAT3 expression in cell lines transfected with miR-125-5p in OSA. ^∗∗∗^represents *P* < 0.001.

**Figure 5:** Validation of molecular targets of miR-123-5p. (a) Differential expression of STAT3 in tumor and normal tissues. (b) Expression of STAT3 in four cell lines of OSA. (c) Expression of drug resistance-associated genes after knockdown of STAT3. ^∗∗∗^represents *P* < 0.001.

**Figure 6:** STAT3 enhances cell viability and reduces apoptosis. (a) CCK8 experiments showed that transfection of miR-125b-5p and STAT3 in complex contributed to increased cell viability. (b) Western blot demonstrated that transfection of miR-125b-5p and STAT3 in complex helped to attenuate apoptosis. ^∗^represents *P* < 0.05; ^∗∗^represents *P* < 0.01; ^∗∗∗^represents *P* < 0.001; ^#^represents *P* < 0.05; and ^###^represents *P* < 0.001.

## Data Availability

The raw data supporting the conclusions of this manuscript will be made available by the authors, without undue reservation, to any qualified researcher.
